The article "Enamel remineralization and repair results of Biomimetic Hydroxyapatite toothpaste on deciduous teeth: an effective option to fluoride toothpaste" was published in 2019. Journal: J Nanobiotechnology.

# Enamel remineralization and repair results of Biomimetic Hydroxyapatite toothpaste on deciduous teeth: an effective option to fluoride toothpaste

**DOI:** 10.1186/s12951-019-0454-6

**Published:** 2019-01-25

**Authors:** Maurizio Bossù, Matteo Saccucci, Alessandro Salucci, Gianni Di Giorgio, Erika Bruni, Daniela Uccelletti, Maria Sabrina Sarto, Giuseppe Familiari, Michela Relucenti, Antonella Polimeni

**Affiliations:** 1 Department of Oral and Maxillo-Facial Sciences, Sapienza University of Rome, Viale Regina Elena 287a, 00161 Rome, Italy; 2 Department of Biology and Biotechnology “Charles Darwin”, Sapienza University of Rome, Piazzale Aldo Moro 5, 00185 Rome, Italy; 3 Department of Aerospace, Electrical and Energy Engineering, Sapienza University of Rome, Via Eudossiana 18, 00184 Rome, Italy; 4 Department of Human Anatomy, Histology, Forensic Medicine and Orthopaedics Section of Human Anatomy Electron Microscopy Unit, Laboratory “Pietro M. Motta” Faculty of Pharmacy and Medicine, University of Rome La Sapienza, Via A. Borelli 50, 00161 Rome, Italy

**Keywords:** Biomimetic nanocrystals, Carbonate-hydroxyapatite, Enamel remineralization toothpaste, Zn-carbonate hydroxyapatite

## Abstract

**Background:**

Dental caries is a recognized worldwide public health problem. Despite being one of the most effective strategies against dental caries, the excessive use of fluorine may result in a potential risk of developing dental fluorosis especially in children under age of six. The purpose of this work is to analyze a fluorine-free toothpaste containing Biomimetic Hydroxyapatite to assess enamel re-mineralizing and repairing properties.

**Results:**

The study was performed in vitro and in vivo, comparing the hydroxyapatite toothpaste with two others toothpaste containing different fluorine concentrations. The coating effect of the micro-structured Hydroxyapatite nanoparticles reintegrates the enamel with a biomimetic film reproducing the structure and the morphology of the biologic Hydroxyapatite of the enamel. As demonstrated, the coating is due to the deposit of a new layer of apatite, which presents fewer particles than the natural enamel, not based on the chemical—physical changes occurring in fluorinated toothpastes. Moreover, it shows resistance to brushing as a consequence of chemical bonds between the synthetic and natural crystals of the enamel.

**Conclusions:**

The use of Biomimetic Hydroxyapatite toothpastes has proven to be a valuable prevention measure against dental caries in primary dentition since it prevents the risk of fluorosis.

## Background

Dental caries is the most common non-communicable chronic disease on a global scale, with a significant impact on the public healthcare expenditure as well as the quality of life of each individual. Epidemiological data indicates that in most industrialized countries the situation is critical, with 60–90% of the children of school age being affected by dental caries. According to the 2015 Global Burden of Disease (GBD) Study, untreated caries in permanent teeth is the most widespread condition among 313 diseases assessed, affecting 2.3 billion people; instead, untreated caries in deciduous teeth has shown a prevalence of 7.8%, affecting 573 million children [1]. An oral health study carried out by the WHO in Italy on children aged 4 and 12, shows a prevalence of caries respectively of 21.6% and 43.1% [2]. Untreated caries in children is associated with conditions such as distress, chronic pain, nutrition and sleep disorder, risk of infection and hospitalization. These issues impact significantly their weight, growth, quality of life. Children’s cognitive development is also hampered due to frequent school absences whose consequences is learning difficulties [3]. The cost increase for treatments must also be taken into account [4, 5]. Caries have a multifactorial etiology, characterized by the loss of nonorganic elements of the tooth`s hard tissues due to the presence of weak organic acids produced by cariogenic bacteria, typically *Streptococcus mutans*, produced by the metabolism of simple carbohydrates introduced by our diet. The increase of acidity in the oral environment triggers the dissolution of hydroxyapatite crystals of the tooth enamel and spreads calcium and phosphate ions [6]. Saliva becomes oversaturated with calcium and phosphate, contributing in the decrease of minerals on the enamel surface, previously demineralized, and increases the resistance to the cariogenic process [7]. In this dynamic process of demineralization and re-mineralization, it is essential to reduce the pathologic factors that increase the chance of dental caries. The use of fluorine as the primary prevention against dental pathologies is widely documented in literature, and its key role is acknowledged since the water fluorination. The ability of fluorine to re-mineralize dental surfaces is widely demonstrated for both permanent and deciduous teeth [8]. For over 50 years it has been recommended to use products based on fluorine and toothpaste represents by far the most common one [9, 10], able to provide higher concentrations of fluorine compared to drinking water. Despite being one of the most effective strategies which led to a drop in caries in industrialized countries [11], it must be taken into account that water fluorination, fluorine supplements in our diet, the use of toothpastes and topical application of fluorine may result in a potential risk of developing dental fluorosis [12]. At an early age, children do not possess full control of the swallowing process and involuntarily ingest toothpaste during the daily oral hygiene practice, resulting in a systematic accumulation of fluorine [13, 14]. Although the use of toothpastes with high concentration of fluorine (1500 ppm) allow greater caries control, using these products on children under 6 years of age increases the chance of fluorosis, which is directly linked to the quantity and concentration of fluorine ingested. Even if statistically, toothpastes with low concentration of fluorine (500 ppm) have not shown a significant effect on caries prevention, they are definitely safer [6]. Current recommendations for children under six indicate the use of toothpastes with at least 1000 ppm of fluorine in pea-sized quantity, under parental supervision [7]. As an alternative to fluorine toothpaste, children under the age of six may use a toothpaste containing biomimetic apatite [15, 16]. Such a toothpaste could be highly recommended, eliminating the potential risk of fluorosis. The purpose of this work is to analyze a fluorine-free toothpaste containing Biomimetic Hydroxyapatite (Zinc-Substituted Carbonate-hydroxyapatite, Microrepair), to assess enamel re-mineralizing and repairing properties as well as the antibiofilm activity against *Streptococcus mutans*. The study was performed *in vitro* and *in vivo*, comparing the hydroxyapatite toothpaste with two others toothpaste containing different fluorine concentrations, in order to understand its interaction with the dental tissues and demonstrating its potential in terms of protecting elements of deciduous teeth.

## Materials and methods

Three different toothpaste were compared: (a) common toothpaste, (b) commercial toothpaste containing fluorine 500 ppm; (c) commercial toothpaste containing fluorine 1400 ppm; (d) toothpaste containing Hydroxyapatite nanocrystal (Biorepair^®^, Coswell S.p.A., Funo, Bologna, Italy). Biorepair^®^ toothpaste was analyzed by means of HR-SEM microscopy (High Resolution Scanning Electron Microscopy). VP-SEM (Variable Pressure Scanning Electron Microscopy) analysis on dental samples treated with different toothpastes was also carried out. Finally antimicrobial properties of Biorepair^®^ were tested. This study was approved by the Ethical Committee at Sapienza University of Rome (no 4681); an informed consent forms were signed by the parents of all patients.

### Biorepair^®^ preparation protocols for HR-SEM

Biorepair^®^ toothpaste was previously characterized as reported by Peetsch et al. [17]. For HR-SEM analysis it was placed on a microscope slide and left in a desiccator for 24 h prior to observation. In order to isolate microRepair^®^ particles from the polymeric phase, to study their morphological features, magnetic stirring and centrifugation were used. These non-invasive techniques do not affect particles morphology at FE-SEM (Field emission scanning electron microscopy) observation. Different protocols of stirring and centrifugation were tested.

Biorepair^®^ toothpaste was dissolved in DI water inside a 250 ml becker and then subject to magnetic stirring at 500 rpm for 20 min. The sample was left overnight to sediment. The supernatant was then retrieved and deposited on Si/SiO_2_ for microscopic analysis (Sample Br). Biorepair^®^ toothpaste was dissolved in DI water inside a 250 ml becker and then subject to magnetic stirring at 500 rpm for 20 min. The resulting solution was left overnight to sediment and successively the particles sedimented on the bottom of the becker were recovered, eliminating the supernatant, and deposited on Si/SiO_2_ (Sample B1). In order to optimize the material to be observed, the toothpaste dissolved in DI water as described in (a) and (b) was further subjected to centrifugation at 4000 rpm for 15 min. The sediment particles were then recovered, eliminating the supernatant, and deposited on Si/SiO_2_ (Sample F1). The sediment obtained in F1 was further diluted and underwent an additional centrifugation at 4000 rpm for 15 min. The sedimented particles were then recovered, eliminating the supernatant, and deposited on Si/SiO_2_ (Sample F2).

### VP-SEM analysis of dental surfaces

Two groups of dental surfaces were observed and compared, the control group (manually treated) and the patient group.

#### Control group

The control group was formed using a selection of 30 primary teeth (first deciduous molars in patients aged between 7 and 10 years). The teeth were extracted as a result of orthodontic treatments or physiological replacements. The procedures were performed at the UOC of Pediatric dentistry Sapienza University of Rome department of Oral and Maxillo-Facial Sciences. Each element, with no sign of cracks on the enamel, was preserved in normal saline and then selected at a cementum-enamel junction level in order to remove the root portion, by means of a numerical control diamond-tipped saw Secotron 200. The surface obtained was then glued onto a polycarbonate plate in order to perform two orthogonal cuts of the crown in each tooth in the mesio-distal and in the bucco-lingual direction, finally obtaining four similar fragments. The glued surface was later lapped in order to remove glue residues. Every quarter of crown of each tooth was covered with composite resin at the edges, joined to a resin cylindrical support, to prevent any contamination. Only the external and occlusal surfaces are free and have been etched with 37% orthophosphoric acid for 1 min in order to reproduce the demineralization that occurs in the oral environment, rinsed at the end with normal saline. The resin support on which the fragments are placed is glued onto the bottom of the cap of the falcon specimen, making the sample easy to brush and preserve in normal saline at the end of every treatment. Each fragment of the same tooth was manually brushed for 15 days three times a day using pediatric toothbrushes for 2 min with four different toothpastes: (a) Neutro-Pasta basic with no active component, (b) commercial toothpaste containing fluorine 500 ppm, (c) commercial toothpaste containing fluorine 1400 ppm, (d) Biorepair^®^. Each section was rinsed and preserved in normal saline solution, renewed every brushing session. To observe enamel prisms, one tooth was also artificially demineralized.

#### Patient group

The patient group was selected by eating and oral hygiene habits similar to the control group. Each patient, aged between 7 and 10 years, was advised to use four different toothpastes (ordinary fluorinated toothpaste, Biorepair^®^, Fluorine 500 ppm, Fluorine 1400 ppm), 3 times a day for 15 days. First deciduous molars were finally extracted from patients selected, similar with the control group, as a result of orthodontic treatments or physiological replacements.

### VP-SEM observation protocol

Samples belonging to both control group and patient group were mounted on aluminium stub without any drying or coating procedure. Samples were observed by Hitachi SU 3500 VP-SEM (6–650 Pa) at operating conditions of 30 Pa and kV ranging from 5 to 10. This particular innovative microscope is equipped with several detectors: secondary electrons detector (SE), ultra variable-pressure detector (UVD), back scattered electrons detector (BSE). This instrument allows teeth observation at variable pressure, humidity and low voltage. If compared with conventional high vacuum SEM, VP SEM works at preferable condition, avoiding sample physical damage due to the effect of high voltage electron beam and high vacuum condition. Moreover, VP-SEM does not requires any dehydration or sputter-coating procedures, that alter natural surface features, and suppresses charge-up phenomenon, typical of non-conductive specimens in high vacuum conditions [17, 18]. The image output used was from the Ultra Variable-Pressure Detector (UVD), a BSE image compo mode was also presented. UVD detects photons generated by the interaction of accelerated secondary electrons with gas molecules in the low vacuum environment of the chamber, so it is particularly suitable to obtain surface information at low vacuum and low accelerating voltages. These working conditions are essential for non-destructive observations on biological, non conductive and vulnerable specimens as teeth. BSE image compo mode in low vacuum means that the image results from the overlapping of images generated by secondary electrons ad back scattered electrons. BSE image compo mode in low vacuum contains information about sample composition, but less topography, that’s why to perform roughness surface analysis we used VP-SEM UVD images, analyzed by Image J roughness analysis plug in [19]. Roughness analysis data were statistically analized by MedCalc© statistical analysis software.

### Microbiological analysis

The bacterial strain used in this work was *Streptococcus mutans* ATCC 25175. It was grown in Brain Heart Infusion broth (BHI, DIFCO) at 37 °C. 1 × 10^7^ cell/ml of a over-night growth culture of *S. mutans* was inoculated in 1 ml of sterile phosphate buffered saline (PBS) with a 5% of toothpaste content and incubated for different times of treatment (30 min, 1 h and 4 h) at 37 °C under gentle shaking. This was done for the commercial toothpaste containing fluorine 1400 ppm and for Biorepair^®^ paste. Even a lower concentration (1%) of Neutro-Pasta basic without active component and Biorepair^®^ paste were tested but for a longer treatment time (4 h at 37 °C). After the exposure, samples were diluted and then spread onto BHI agar plates, following incubation at 37 °C. The capacity of the bacteria to form colonies was measured by counting the number of colony forming units (CFU). Results were compared with the control sample, represented by untreated solution. Furthermore, the biofilm produced by the *S. mutans* on the sections of the deciduous teeth treated with different toothpastes was analyzed accordingly [20]. Briefly, each fragment of tooth was subjected to sterilization by UV rays and then placed in a 12-well microtiter plate. An overnight culture of *S. mutans* was diluted to 5 × 10^6^ cells/ml into BHI with 5% sucrose and 3 ml of such bacterial suspension was added to each well. Biofilm was grown on teeth for 24 h at 37 °C under static conditions. After growing, a Crystal Violet (CV, Sigma) assay was performed to quantify biofilm formation on teeth samples. Afterwards, teeth samples were washed twice with sterile water, fixed for 15 min at 65 °C and then stained with 0.3% CV for 15 min. Several washings with sterile water were done and teeth were air-dried and lastly photographed. Finally, 96% ethanol was used to elute CV bound to teeth biofilm and absorbance at 600 nm was then read for CV quantification. The percentage of biofilm formation was compared to the one found on the teeth brushed with Neutro toothpaste, the silica base, used as control.

### Statistical analysis

All experiments were performed at least in triplicate. Data are presented as mean ± SD. The statistical significance was determined by one or two-way ANOVA analysis coupled with a Bonferroni post-test (GraphPad Prism 5.0 software, GraphPad Software Inc., La Jolla, CA, USA), and defined as *P < 0.05, **P < 0.01, and ***P < 0.001.

### Roughness measurement and statistical analysis

In order to provide both qualitative and quantitative results, that allows us to accurately compare different toothpaste effect, for each treatment (common toothpaste, fluorine toothpaste 500, fluorine toothpaste 1400, Biorepair^®^) we analyzed ten micrograph at 500× magnification by means of Image J roughness analysis plug in [21]. The roughness parameter that we considered was Rq (Rq: profile root mean square deviation, it indicates the root mean square value of the ordinates values within a sampling length). Rq values in each treated group were statistically analyzed by Med Calc© statistical software (Ostend, Belgium). Summary statistics (in order to asses normal distribution of data) and then t- test (in order to determine statistical differences between groups) were performed.

## Results

### HR-SEM analysis

A preliminary analysis of Biorepair^®^ clearly shows microstructures covered with basic matrix (Fig. 1). Different sample preparation protocols allowed to improve particles observation. In both Sample Br and B1 aggregated particles were visible in the sediment and in the supernatant. The size of those particles ranges from 50 to 100 nm (Fig. 2a, b). Using centrifugation the microfillers recovered from the sediment of Sample F1 appear as micro-agglomerates of particles (Fig. 2c, d). The size of nanostructured micro-agglomerated is approx. 5 µm and the size of the fine nanostructure characterizing the micro-particles ranges from 50 to 100 nm. Through additional dilution of the sediment obtained in F1, Sample F2 presents micro-agglomerates of approx. 20 micron and the size of the fine nanostructure of the micro-particles ranges from 50 to 100 nm (Fig. 2e, f).

**Fig. 1:** SEM Image of desiccated Biorepair^®^ toothpaste

**Fig. 2:** Different sample preparations. SEM images of sample Br and B1 (**a**, **b**), sample F1 (**c**, **d**) and sample F2 (**e**, **f**) at different magnifications

### VP-SEM dental surface analysis

#### Imaging of the artificially demineralized tooth

At a low magnification of 500× dental surface shows a cribrous aspect. At higher magnification (5000×), a honeycomb structure appears and Hydroxyapatite prisms are visible (Fig. 3).

**Fig. 3:** SEM micrograph of the artificially demineralized tooth (**a** ×500, **b** ×5000)

#### Imaging of control group and patient group

In Fig. 4 effect of neutral toothpaste on both groups is illustrated. The surfaces of both samples show a great deal of similarities. At low magnification (500×) some slightly worn layers, with a visible superficial roughness are showed. At higher magnification (5000×) disaggregated particles, with heterogeneous shape and dimension, appear to be fairly uniformly distributed on tooth surface (Fig. 4). In Fig. 5a, b effect of Fluorine 500 toothpaste on both groups is illustrated. Fluorine 500 ppm toothpaste treatment does not present major changes in both groups with respect to neutral toothpaste. Surfaces present a cribrous layer, uneven, with a worn out appearance and visible crater-like spaces, which can be better observed at higher magnification (Fig. 6a, b). In Fig. 5c and d effect of Fluorine 1400 toothpaste on both groups is illustrated. The treatment with Fluorine 1400 ppm leaves a layer of material on dental surface which covers in part surface erosion craters. Anyway dental surface is not smooth, it still preserves a higher degree of roughness as well as an unequal distribution of the material. The material is laid down in a fine granulation with uneven aspect. Sometimes aggregated material is visible (Fig. 6c, d). Also in this case no differences between control and patient group is visible. In Fig. 5e and f effect of Biorepair^®^ toothpaste on both groups is illustrated. At low magnification (500×) Biorepair^®^ treated surfaces, appear covered by a uniform, very smooth and fine layer of material. Enamel micro-cavities are filled, even though their borders are visible (but their aspect is very blunt). At higher magnification (5000×) deposit, homogeneity is clearly visible, no heterogenous granulations were observed (Fig. 6e, f). This suggests a levelling property that mitigates the superficial roughness and ensures an even and uniform coverage of the dental surface. Biorepair^®^ treatment recalls the smoothing effect of the face powder. Both patients and control samples, shows same results. In Fig. 7 effect of Biorepair^®^ treatment after common toothpaste treatment is showed. As an additional test to asses Biorepair^®^ treatment results, we used 2 deciduous teeth from common toothpaste treated patient group. One tooth was extracted and analyzed without any additional treatment, ensuring that the patient has used common pediatric fluorinated toothpaste (Fig. 7a). The second was extracted and analyzed after 15 days of Biorepair^®^ manual brushing (Fig. 7b). Before and after treatment difference is remarkable. As a matter of fact, before treatment, pictures shows presence of scratches and groves (Fig. 7a, c). After treatment with Biorepair^®^, figures reveal the almost total absence of scratches and groves, which are filled and levelled due to microRepair^®^ particles (Fig. 7b, d). The surface is smooth and homogeneously repaired thanks to the coating action of the material.

**Fig. 4:** SEM images of neutral toothpaste treatment: control group dental surfaces (**a**, **c**) patient group dental surface (**b**, **d**). Magnification ×1000 **a**, **b**. Magnification ×5000 **c**, **d**. In **b** flattened cells of the oral epithelium are showed (arrow)

**Fig. 5:** SEM images (magnification ×500) of different treatments on dental surfaces. Fluorine 500 ppm toothpaste in control group (**a**) and patient group (**b**); Fluorine 1400 ppm toothpaste in control group (**c**) and patient group (**d**); Biorepair^®^ toothpaste in control group (**e**) and patient group (**f**). In **f** flaked off cells from the patient's oral epithelium are present (arrow)

**Fig. 6:** SEM images (magnification ×5000) of different treatments on dental surfaces. Fluorine 500 ppm toothpaste in control group (**a**) and patient group (**b**); Fluorine 1400 ppm toothpaste in control group (**c**) and patient group (**d**); Biorepair^®^ toothpaste in control group (**e**) and patient group (**f**)

**Fig. 7:** Biorepair^®^ toothpaste additional test SEM images of **a** control surface before treatment with a common fluorinated toothpaste and **b** after treatment with Biorepair^®^; **a** and **b**, magnification ×500, **c**, **d** magnification ×1000

### Roughness analysis results

Rq values of differently treated surfaces resulted normally distributed (Table 1). T-test result listed below (Table 2) show significative differences among all groups with the exception of neutral vs fluorine 500. The statistical analysis results of Rq values demonstrate that there is no statistically significant difference between Fluorine 500 toothpaste and common toothpaste (P = 0.0630); toothpastes effects are equivalent. A statistically significant difference exists when Fluorine 500 toothpaste is compared to Fluorine 1400 toothpaste (P = 0.0157) and when Fluorine 1400 toothpaste is compared to Biorepair^®^ toothpaste (P = 0.0224), in these cases we can say that toothpastes have different repairing properties. An high statistically significant level is obviously reached when the effect of common toothpaste is compared to that of Fluorine 1400 (P = 0.0001), and with that of Biorepair^®^ (P < 0.0001). Being Fluorine 500 toothpaste effect similar to that of neutral toothpaste, a high statistically significant level is reached also when Fuorine500 is compared to Biorepair^®^.

**Table 1:** Data of roughness

Rq values	Common toothpaste	Biorepair	Fluorine500	Fluorine1400
Sample size	10	10	10	10
Lowest value	162.3410	85.3950	148.2470	106.6610
Highest value	187.5240	144.7160	194.2820	168.5540
Arithmetic mean	175.1830	123.4368	163.8533	144.4307
95% CI for the arithmetic mean	168.7841 to 181.5819	108.7276 to 138.1460	152.6110 to 175.0956	132.3918 to 156.4696
Median	176.8020	131.3735	160.3755	146.0630
95% CI for the median	166.1845 to 183.6649	100.4502 to 140.4814	150.4373 to 179.1781	136.2510 to 156.6117
Variance	80.0134	422.7956	246.9807	283.2233
Standard deviation	8.9450	20.5620	15.7156	16.8292
Relative standard deviation	0.05106 (5.11%)	0.1666 (16.66%)	0.09591 (9.59%)	0.1165 (11.65%)
Standard error of the mean	2.8287	6.5023	4.9697	5.3219
Coefficient of Skewness	− 0.04060 (0.9511)	− 0.9807 (0.1488)	1.0164 (0.1352)	− 1.0634 (0.1189)
Coefficient of Kurtosis	− 1.5119 (0.1600)	− 0.4064 (0.8836)	0.01875 (0.8299)	2.3140 (0.1164)
D’Agostino− Pearson test for normal distribution	Accept normality (0.3719)	Accept normality (0.3488)	Accept normality (0.3202)	Accept normality (0.0864)

**Table 2:** Indipendent t test among treated samples

	Test statistic t	Degrees of freedom	Two-tailed probability significative P < 0.05
Rq_common Vs Rq_Fluorine500	− 1.981	18	0.0630
Rq_common Vs Rq_Fluorine1400	− 5.102	18	0.0001
Rq_common Vs Rq_Biorepair	− 7.298	18	0.0001
Rq_Fluorine500 Vs Rq_Fluoine_1400	− 2.667	18	0.0157
Rq_Fuorine500 Vs Rq_Biorepair	− 4.938	18	0.0001
Rq_Fluorine_1400 Vs Rq_Biorepair	− 2.499	18	0.0224

### Antimicrobial and antibiofilm assays

*Streptococcus mutans* has been identified as the main etiologic cause of dental caries [22] and growing interest is focused on the development of suitable materials, such as toothpastes, able to kill or inhibit this bacterium and, thus, to control the pathologic conditions. Microbiological tests performed on the toothpastes showed a very similar resistance of bacterial cells exposed to a 5% aqueous solution of the fluoride-based toothpaste or the Biorepair^®^, compared to the treatment with water (UT) as shown in Fig. 8. As the time of the exposure increase the vitality rate decreases, with a similar antimicrobial power in both toothpastes (Fig. 8a). Notably Biorepair^®^ also exhibited higher anti-Streptococcus activity at 1% (w/v) when incubated with bacterial cells for 4 h (Fig. 8b). Due to the anti-Streptococcus action, it was evaluated the ability of the Biorepair^®^, to inhibit biofilm adhesion and growth on deciduous teeth samples. To this purpose, the deciduous teeth were treated with the different toothpastes 3 times a day for 15 days. The results of the assessment of the biofilm produced by *S. mutans* on the sections of the fragments of deciduous teeth indicate that the action of Biorepair^®^ can be almost identical to other toothpastes. The analysis was performed by the Crystal Violet (CV) method that allows the determination of biofilm mass (Fig. 8c). This can be also visualized by the pictures of CV stained fragments deciduous teeth surfaces treated with the different products, as indicated (Fig. 8d).

**Fig. 8:** **a** CFU results of *S. mutans* treated and not with 5% toothpastes in saline solutions at various times. Bacterial survival is expressed in CFU rate compared to untreated one. Statistical analysis was performed by two-way analysis of variance (ANOVA) method coupled with the Bonferroni post-test. Different letters indicate different statistical significances. **b** *S. mutans* cell survival after treatment for 4 h in saline solutions with 1% of toothpastes content. Error bar indicates standard deviation. Statistical analysis was performed by one-way ANOVA method coupled with the Bonferroni post-test (**P <* 0.01* compared to the control). **c** Biofilm biomass analysis on CV stained deciduous teeth. Data are expressed as percentage of biofilm formation relative to control teeth brushed with Neutro-pasta toothpaste. Histograms are the mean of three independent experiments. Error bars indicate SD and statistical analysis was performed by one-way ANOVA method coupled with the Bonferroni post-test (ns not significant). **d** Photographs of teeth brushed with the different types of toothpaste and stained with CV after *S. mutans* biofilm growing

## Discussion

Elements of deciduous teeth present thinner enamel, nearly half the size compared to permanent teeth [23]. Moreover, the enamel is thinner and more fragile, therefore prone to fractures due to a lower level of mineralization, which had a negative impact on mechanical properties [24]. All this can have a greater impact and a rapid development of caries and erosion on deciduous teeth [25, 26]. An early non-invasive treatment of incipient lesions through remineralization of the enamel surface is one of the constantly evolving fields of research. The rapid growth of biomaterials and nanotechnologies fostered the development of innovative products with advanced bio-reactive and biomimetic properties. Furthermore, nanostructured materials have a better performance compared to their counterparties containing micro-dimensioned particles, due to their higher surface/volume ratio. Biorepair^®^, Biomimetic Hydroxyapatite-Carbonate based and synthesized with “bottom up” nanotechnology processes [27], is made of nanostructured micro-particles, having average size in the range of 5–20 µm and fine nanostructure ranging from 50 to 100 nm (Fig. 2). The effect of the application remineralized toothpaste of latest generation was observed through scanning electron microscopy (SEM), compared to the effect of fluorinated toothpaste on elements of deciduous teeth, in vitro and in vivo, prior to artificial demineralization of the enamel with orthophosphoric acid. The treatment with 1400 ppm fluorine toothpaste (Fig. 5c, d) clearly shows the remineralizing potential, with changes on a morphological level of the surface, maintaining roughness and homogeneous appearance. His feature is deeply remarked in samples treated with 500 ppm fluorine toothpaste, where the surface is even more cribriform (Fig. 5a, b). The results are in line with several studies indicating low protection levels in toothpastes with low fluorine content compared to those with higher concentrations [28–30]. Although the validity of with low doses of fluorine is controversial, it lowers the risk of fluorosis by accidental ingestion of the product [31, 32]. Studies on the samples treated with Biomimetic Hydroxyapatite toothpaste show a homogeneous surface, in which the roughness of the demineralized enamel are repaired and smoothly leveled. During the years 2010–2013 Orsini et al. produced several clinical randomized trials with promising results demonstrating the efficiency of Biomimetic Hydroxyapatite nanocrystals toothpaste in decreasing dentine hypersensitivity and promote a re-mineralizing mechanism [33, 34]. These in vivo morphological and chemical physics studies may partially explain the beneficial effect of Biomimetic Hydroxyapatite nanocrystals toothpastes in diminishing dentine hypersensitivity, for the fact that the deposition of a synthetic Hydroxyapatite nanocrystals coating may produce a re-mineralizing/repairing effect on the enamel surface, in teeth treated with toothpaste containing Hydroxyapatite nanocrystal [35, 36]. Therefore, as demonstrated by Lelli et al. the re-mineralizing process of such toothpaste can also be confirmed in vivo [37].

Although our study has been carried out on dental elements of the deciduous series the results achieved are consistent with the aforementioned trials and confirm that the effect can produce a biomimetic coating on the enamel surface also in deciduous teeth. Indeed, the coating effect of the nanostructured Hydroxyapatite micro-particles reintegrates the enamel with a biomimetic film reproducing the structure and the morphology of the biologic Hydroxyapatite of the enamel (Fig. 5e, f). As demonstrated, the coating is due to the deposit of a new layer of apatite, which presents fewer particles than the natural enamel, not based on the chemical–physical changes occurring in fluorinated toothpastes. Moreover, it shows resistance to brushing as a consequence of chemical bonds between the synthetic and natural crystals of the enamel [38]. This feature has been highlighted by our study on elements of deciduous teeth extracted from the same patient, in which the first element indicated the presence of grooves despite the use of fluorinated toothpaste for daily dental care (Fig. 7a, c). The second element was analyzed, additional to the first extract, after a 15-day treatment with Biorepair^®^ showed a progressive filling of the damaged enamel (Fig. 7b, d). The results obtained with micrograph scanning are validated by the roughness analysis carried out on the samples which show a significant difference in roughness between the samples treated with fluorinated toothpaste and those treated with Biorepair^®^. Microbiological tests on toothpaste and samples of deciduous teeth have proven that Biorepair^®^ possess anti-bacterial properties against Streptococcus mutans cells and the ability to inhibit the biofilm production, similar to other fluorinated toothpastes. The impact on bacterial adhesion was investigated in situ since bio-adhesion processes under in vivo and in vitro conditions can differ considerably [39]. Only in situ or in vivo experiments give optimal insight into the interactions of oral health care devices with the dental hard tissues and the oral biofilm. These data highlights for the first time the advantages of Biorepair^®^ in pediatric age in comparison with fluoride-based preparations.

Indeed, the excessive intake of fluoride during the maturation of the enamel for children under age 6, can cause an alteration in the mineralization of the tooth [39].

In vitro studies have shown that the inhibition of the demineralization of synthetic carbonate hydroxyapatite can be expressed with a logarithmic function of the fluorine concentration in the surrounding solution [35]. The systemic intake of fluoride during tooth formation has been shown to be effective in preventing caries or in inhibiting the demineralization of tooth apatitis; however, according to the opinion of the NDA Panel of the European Food Safety Authority, intake of 0.1 mg of fluorine per kg body/day in children up to the age of 8 may be considered as the limit dose, below which no fluorosis of permanent teeth may occur [36–38].

While a mild dental fluorosis is not immediately visible, a moderate fluorosis can be easily appreciated and is characterized by white spots and opaque streaks and irregularities on the surface of the teeth [40].

In any case, it is important to consider that fluorine-containing water; fluorine supplements in diets, fluoride toothpastes and local fluoride applications have been identified as a source of enamel fluorosis. In addition the fluorine present in toothpastes, despite being known for its anti-caries properties, becomes toxic if ingested at high concentrations, especially in children, in relation to weight difference [41, 42]. The minimum dose that can cause signs of toxicity has been calculated in 5 mg of fluorine/kg of body weight [43]. Finally although the effects of biomimetic toothpaste are so considerable, a long-term studies of its properties is needed.

## Conclusion

The use of nanostructured micro-particles in Biomimetic Hydroxyapatite toothpastes has proven a high potential of remineralization of the enamel of deciduous teeth, becoming a valuable prevention measure against cavities especially for high-risk individuals such as children before the schooling age, since it prevents the risk of fluorosis.
